# Integration of Global and Local Features for Specular Reflection Inpainting in Colposcopic Images

**DOI:** 10.1155/2021/5401308

**Published:** 2021-07-27

**Authors:** Xiaoxia Wang, Ping Li, Yuchun Lv, Huifeng Xue, Tianxiang Xu, Yongzhao Du, Peizhong Liu

**Affiliations:** ^1^College of Medicine, Huaqiao University, Quanzhou, Fujian 362021, China; ^2^Department of Gynecology and Obstetrics, The First Hospital of Quanzhou, Quanzhou, Fujian 362000, China; ^3^Cervical Disease Diagnosis and Treatment Health Center, Fujian Provincial Maternity and Children's Hospital, Affiliated Hospital of Fujian Medical University, Fuzhou, Fujian 350001, China; ^4^College of Engineering, Huaqiao University, Quanzhou, Fujian 362021, China

## Abstract

**Objective:**

To explore an inpainting method that can balance texture details and visual observability to eliminate the specular reflection (SR) regions in the colposcopic image, thus improving the accuracy of clinical diagnosis for cervical cancer.

**Methods:**

(1) To ensure smoothness, Gaussian Blur and filling methods are applied to the global image. (2) Striving to preserve the anatomical texture details of the colposcopic image as much as possible, the exemplar-based method is applied to local blocks. (3) The colposcopic images inpainted in the previous two steps are integrated, so that important information of non-SR regions is preserved based on eliminating SR regions.

**Results:**

In the subjective visual assessment of inpainting results, the average of 3.55 ranks first in the five comparison sets. As to the clinical test, comparing the diagnosis results of 6 physicians before and after eliminating SR regions, the average accuracy of two kinds of classifications increased by 1.44% and 2.03%, respectively.

**Conclusions:**

This method can effectively eliminate the SR regions in the colposcopy image and present a satisfactory visual effect. *Significance*. As a preprocessing method for computer-aided diagnosis systems, it can also improve physicians' accuracy in clinical diagnosis.

## 1. Introduction

According to World Health Organization (WHO) Global Cancer Statistics Report in 2018, cervical cancer ranked fourth in both incidence and mortality [1]. The latest statistics from the US indicate that cervical cancer remains the second leading cause of cancer deaths among women aged 20 to 39 years old [2], posing a severe threat to women's health. Clinical studies have confirmed that persistent high-risk human papillomavirus virus (HR-HPV) infection is the leading cause of the development of cervical cancer. It takes years or even decades for patients with persistent HR-HPV infection to develop from HPV infection to cervical cancer, and they also experience a long precancerous stage (CIN1, CIN2, and CIN3) [3], during which clinicians can early detect, treat, and remove the affected tissues to prevent cervical cancer [4]. Despite the continued development of the HPV vaccine, its popularity cannot meet current needs due to its price and geographical differences. Therefore, a large-scale and standardized cervical cancer screening program for the general population is one of the most effective ways to reduce the incidence and mortality of cervical cancer.

Currently, there are three mainstream screening methods: pap cytology, colposcopy, and biopsy [5]. Among them, colposcopy has become a critical assistant tool for cervical cancer screening due to its simple operation and low cost. Colposcopy is an optical instrument that can adjust the light source to penetrate the tissue, magnify the cervical epithelium and blood vessels, and discover potential cervical lesions and evaluate them. Therefore, when the light from the camera flash irradiates the cervical tissue during the colposcopy, some specular reflection (SR) regions often appear in colposcopic images due to the presence of physiological mucus on the surface of the cervical tissue [6]. As shown in Figure 1, in the colposcopic image, these SR regions have similar characteristics as the acetic white (AW) regions [7], which are essential tissue changes in lesion regions after the application of acetic acid. In addition, if the surface color, texture features, and saturation of the cervical tissue are weakened, the images will show high brightness and low saturation. It will result in the uneven appearance of cervical epithelial tissue and even complete loss of surface information. This phenomenon also interferes with the recognition, segmentation, and classification of cervical lesions by the computer, thereby reducing the accuracy of the cervical intelligent assistant diagnosis system. In practical applications, the preprocessing of the colposcopic image to eliminate SR regions has become an essential task for the intelligent diagnosis of cervical lesions.

## 2. Related Work

At present, many researches on the intelligent diagnosis of colposcopic images do not consider the impact of SR regions [8, 9] or just perform simple threshold processing to eliminate reflective pixels. Only a few studies on the recognition and classification of cervical lesions have considered the interference of SR regions.

Two main directions in the research on SR regions' elimination in natural images: one is the dichromatic reflection model (DRM) based on physical methods to automatically eliminate SR regions [10, 11]. It defines the color as a linear combination of object color and highlight color [12]. Another is to use polarization filters to determine SR regions [13] and then performs analysis and statistics based on the integration of multiview color and polarization information.

Since the colposcopic image contains many regions with similar colors but different intensities and textures [14], the above method cannot be fully applied to eliminating SR regions of the colposcopic image. The problem of SR regions has always been a bottleneck restricting the development of automatic extraction algorithms in the colposcopic image.

Most researchers have explored different color spaces. Van et al. [15] expressed the pixel distribution in the image as a Gaussian mixture model in the RGB color space and then distinguished SR pixels and non-SR pixels, while Praba et al. [16] performed Gaussian mixture modeling in the HIS space. Langer et al. [17] and Das et al. [18–20] performed adaptive threshold detection in RGB color space. The former mainly used the R channel, but the latter used the intersection of the three channels. Then, the smoothest interpolation and filling were performed, respectively, by the Laplacian equation. Gordon et al. [21] detected high-brightness and low-saturation regions with fixed thresholds and selected SR candidate regions to continuously refine the pixel range in the S-V space mapped from HSV color space. Zimmerman et al. [14] also adopted the same mapping space but loosened the threshold to determine SR regions and non-SR regions more reasonably. Besides, they added the Gaussian distribution description to them and then used the iterative filling method to repair. This method requires high prior knowledge and has difficulties in actual operation. Meslouhi et al. also detected SR features in HSV color space initially [22] but later converted to planar XYZ color space, where SR regions were effectively detected by a simple automatic luminance-chromaticity comparison [23]. Here, the DRM described previously was applied. As for the inpainting, they introduced a multiresolution inpainting technique (MIT), which fully considers the different levels of details in a colposcopic image, but the method's stability needs to be verified. Kudva et al. [24] innovatively combined the SR features of HSV, RGB, and Lab color spaces to detect SR regions. Their results were stable and accurate, but the repair method was not precise.

It is worth noting that colposcopic images have many similarities with other endoscopic images, so some standard research methods can be applied to the problem of eliminating SR regions in the colposcopic images. Colonoscopy [25], thoracoscopy [26], laparoscopy [27], and more researches on eliminating SR regions in these images [28, 29] can be used for reference. In the report of Wang et al. [30], they used Arnold's method [25] in colonoscopy images and combined it with the exemplar-based method to eliminate SR regions in colposcopic images, showing better effect.

There is no ground truth without SR regions in the endoscopic image. The irregular distribution of SR pixels makes accurate manual segmentation time-consuming and labor-intensive. And manual annotation is highly dependent on experts, which increases the difficulty of quantitative analysis of the results related to SR regions elimination and limits the application of deep learning in this study, so there are relatively few studies on deep learning for eliminating SR regions in these images [31, 32].

Overall, eliminating SR regions in colposcopic images focuses on the extraction and detection of luminance and chrominance features in different color spaces, and inpainting methods are used to eliminate them. However, these methods fail to effectively balance the visual visibility and detailed preservation to better meet the subsequent processing by computers and clinical diagnosis.

This paper is a further study based on our previous studies [30]. We propose a method to eliminate SR regions based on the integration of global and local features in colposcopic images, which solves the problem that SR regions cannot be wholly eliminated to retain the texture as much as possible. Moreover, through integrating global and local information, the overall visual observability of images is enhanced.

In the experimental part, we thoroughly investigate our method and test its performance from different angles. The results show that this method can better eliminate SR regions in colposcopic images and improve clinicians' diagnostic accuracy. The contributions of this paper are summarized as follows:

1. We comprehensively consider the preservation of texture details and the overall visual observability after eliminating SR regions
2. We propose a method to eliminate SR regions based on integrating the global and local information of the colposcopic image

## 3. Materials and Methods

Since SR regions of colposcopic images are similar to AW regions, it is not easy to directly eliminate them from chromaticity. Researchers usually detect SR regions by brightness and refine the detection by combining absolute pixels and relative pixels. However, when the detection is good, the inpainting often causes the overall image to be excessively smooth. The other way is to consider the texture details of colposcopic images, but the elimination of SR regions is incomplete, resulting in remaining highlight speckle. These two methods are not sufficiently successful in terms of visual observability. When the details of the lesion area are strictly required in clinical diagnosis, they will interfere with the physicians. With all of the above, we combine Arnold's method [25] with the exemplar-based method to eliminate SR regions of colposcopic images. At first, the original colposcopic image is smoothed by the global application of Arnold's method. Then, the colposcopic image is reconstructed after subblocking locally using the exemplar-based method to eliminate SR regions of each block finely. Finally, two images obtained in the previous steps are integrated. The overall process of our method is shown in Figure 2.

### 3.1. Preprocessing

Besides the cervical region diagnosed by physicians, there is other information in colposcopic images, including vaginal walls and other noncervical anatomy, tools (such as speculum and swabs), textual marks, and other marks superimposed on film. The elimination of SR regions is mainly aimed at the cervical region, so our SR region inpainting method is more meaningful on the preliminary preprocessing of original images.

Our data set is prenormalized. Most of the noncervical areas in original colposcopic images are trimmed, and all images are resized to a size of 224 × 224 for the elimination of SR regions. In addition, to further understand whether there is a difference in images with different grades of the cervical lesion after eliminating SR regions, our data set is classified by lesion grade, and the final data sample is shown in Figure 3.

### 3.2. Stage 1: Global Processing

In the global processing, we aim at fine detection and smooth filling by learning from the method of automatic segmentation and inpainting of SR regions in colonoscopy images proposed by Arnold.

Arnold [25] proposed that, based on threshold segmentation of color images to detect SR regions, the nonlinear filtering method is used to divide the highlight pixels into two categories: significantly strong and slightly nonstrong. More accurate detection is performed gradually to avoid the influence of the background brightness. Here, according to the characteristics of high brightness and low color saturation in SR regions of colposcopic images, YUV color space transformation is performed on the image before the original algorithm to obtain the high-brightness component *Y* (*C*_*Y*_). Then, SR pixels are roughly and finely detected in two modules. The overall detection process of this part is shown in Figure 4. Refer to literature [25] for specific methods.

In Arnold's method [25], the gradient feature is used to limit bright non-SR regions. For colposcopic images, SR regions are usually small bright spots, while AW regions are larger white patches. Thus, to prevent certain AW regions from being recognized as SR pixels, we mainly limit the final detection regions based on the size and the brightness threshold.

For inpainting, Arnold eliminates SR regions from two levels [25]. In the first, within a certain distance of the detected edge, all the detected SR regions are replaced by the centroid color of the pixel to obtain a new modified image. Then, the modified image is filtered using the Gaussian kernel (*σ* = 8). Finally, a robust and smooth image without SR regions is output. For the second level, a smooth weighted mask is achieved by adding a nonlinear attenuation over the contour of SR regions.

As mentioned in this literature, the larger SR regions in the image will be very blurred vision due to Gaussian Blur. For the diagnosis of colposcopic images, the requirements for texture details are strict, so if such a large blurred area appears, it will have a terrible effect in clinical practice. To solve this problem, we will introduce the exemplar-based method in the local processing, getting better texture details.

### 3.3. Stage 2: Local Processing

Local processing is mainly aimed at excessive smoothness and lack of texture details after global processing. In the previous work, we used the exemplar-based method proposed by Criminisi et al. [33] and found that this inpainting method can effectively inpaint the texture details in SR regions of colposcopic images. Therefore, we still use the exemplar-based method in this stage to balance the oversmoothing problem.

The distribution of SR regions in colposcopic images is random and uncertain. If we want to eliminate the SR region locally, the simplest solution is to block the overall image and then detect and inpaint SR regions in each block. The image is effectively processed in this way, and blocks without SR regions can be directly skipped, which reduces the time consumption to a certain extent. For the block with SR regions, the proportion of SR regions in the block is larger than the original proportion in the global image. Fortunately, the exemplar-based method works well for such a relatively large area. In addition, when inpainting SR regions in each block, the interference from other global information is less, the confidence is higher, and the processing of texture detail is better. Next, we will elaborate on the detection and inpainting methods in local processing in detail.

#### 3.3.1. SR Regions Detection

We require fine detection in the global processing, but our primary goal is to preserve the texture details of the image in the local processing. Therefore, we do not require precision in detecting SR regions in this part, and we require the texture details to be continuous as much as possible after inpainting. This can improve the visual observability of the colposcopic image. Based on the above considerations and the time consumption, we choose a method that uses the color characteristics of SR regions [23].

Firstly, image enhancement is performed. Since the chromaticity difference between SR regions and AW regions in the colposcopic image is small, we target the chromaticity enhancement in the HSV color space. This nonlinear filter is defined as follows:

(1) $$\begin{array}{c} \left(\begin{array}{c} R^{\prime }\\ G^{\prime }\\ C^{\prime } \end{array}\right)=\left(1-S\right)\left(\begin{array}{c} R\\ G\\ C \end{array}\right)=\frac{\min\left(\text{R},\text{G},\text{B}\right)}{\max\left(\text{R},\text{G},\text{B}\right)}\left(\begin{array}{c} R\\ G\\ C \end{array}\right). \end{array}$$

Then, the pixel luminance (*y*) and the color luminance of the entire image (*Y*_global_) are compared, and the set of pixels meeting the following conditions is defined as SR regions for local detection:

(2) $$\begin{array}{c} y>=\omega Y_{\text{global}}=\omega \frac{Y}{X+Y+Z}. \end{array}$$

Here, we give *Y*_global_ a coefficient with the value of *ω* because we do not focus too much on the small highlight pixels in the local processing, but rather inpaint the relatively large SR regions to present an excellent visual effect. Such a process of increasing the brightness threshold also shortens the subsequent inpainting time. The selection of this coefficient will be specified in the experimental section.

#### 3.3.2. Inpainting

The image inpainting algorithm based on the exemplar-based method uses the pitch as the basic unit. It uses a pixel value and a confidence value to represent the centre pixel of this pitch. After giving a priority value to it, the filling order is determined by the weight value. The best matching pitch is based on a certain matching principle to fill the texture and structure information.

The basic model of the exemplar-based method to inpaint SR regions in the colposcopic image is shown in Figure 5. Here, *I* represents the whole image, Ω is the region to be inpainted, *∂*Ω is its boundary, and the pixel *p* is a point on the *∂*Ω boundary. Ψ_*p*_ is a rectangular neighborhood centred on the point *p*. Φ = *I* − Ω is the non-SR regions.

The inpainting process is as follows:

(1) Determine the boundary of the SR region in the colposcopic image. This can provide the necessary initial information to make the inpainting gradually move from the boundary to the centre.
(2) Calculate the priority of the target pixel *p*. It aims to determine the pitch to be inpainted in the SR region. The calculation formula is as follows:
  (3) $$\begin{array}{c} P\left(p\right)=C\left(p\right)D\left(p\right). \end{array}$$
*C* (*p*) is the confidence item used to measure the completeness of the information in the neighborhood of pixel *p*. A more significant value indicates that the neighborhood of pixel *p* contains more available information. *D* (*p*) is the data item used to measure the location of pixel *p*. The greater the value is, the closer pixel *p* is to the decisive edge. The pitch with a higher priority value and the continuous edge will be filled in earlier to preserve the texture and structure information in SR regions.
The confidence item and data item are expressed as follows:
  (4) $$\begin{array}{c} C\left(p\right)=\frac{\sum_{q\in \psi_{p}\cap \left(1-\Omega \right)}C\left(p\right)}{\left|\psi_{p}\right|}, \end{array}$$
  (5) $$\begin{array}{c} D\left(p\right)=\frac{\left|\nabla I_{p}^{⊥}\cdot np\right|}{\alpha }. \end{array}$$
In the formula, |*Ψp*| is the area of *Ψp*, *α* is the normalization factor, *n*_*p*_ is the standard unit vector of the pixel *p* in the boundary direction, and ⊥ represents the orthogonal operator.
(3) Select the block that best matches the SR region in the known region Φ of the colposcopic image and fill it. According to the Sum of Squared Difference (SSD) matching principle, find the most similar pitch to copy its structure and texture information. The filling result is defined as
  (6) $$\begin{array}{c} \psi_{\hat{q}}=\arg_{\psi q\in \Phi }\min\;d\left(\psi_{\hat{p}},\psi q\right). \end{array}$$
Here, $d\left(\psi_{\hat{p}},\psi_{q}\right)$ is the sum of the squares of the differences between the corresponding pixel values in the two pitches, i.e., the relative distance. The pitch $\psi_{\hat{q}}$ with the smallest distance is selected as the best matching pitch of $\psi_{\hat{p}}$, and the known relevant information in $\psi_{\hat{q}}$ is filled into the position of the SR region in the pitch $\psi_{\hat{p}}$.
(4) Update the confidence value of the corresponding pixel in the SR region. The pixel confidence values $C\left(\tilde{p}\right)$ of the filled parts of the pitch $\psi_{\hat{p}}$ are all replaced by the confidence value $C\left(\tilde{p}\right)$ at the centre point $\hat{p}$ of the pitch. The above steps are continued to be repeated after filling until all SR regions are finally eliminated.

### 3.4. Stage 3: Integration

After the first and second stages, two images focusing on global smoothing and local texture are obtained. The work of this stage is to integrate them effectively.

The colposcopic image is a color image with R, G, and B color channels. If these two images are simply added linearly in the RGB color space, the desired visual effect cannot be achieved. On the contrary, the noise information introduced in the previous inpainting process will be amplified. Therefore, we continue to analyze the colposcopic image itself and find a breakthrough in terms of luminance-chromaticity. At first, both images are converted to the HSV color space, which also contains three components, i.e., Hue (*H*), Saturation (*S*), and Value (*V*). Such color space is more similar to the way humans perceive colors. Then, we compare the three-component values of each pixel in the two images and reserve pixels that meet the following conditions:

(7) $$\begin{array}{c} \left\{\begin{array}{c} H_{\text{new}}=\max\left(H_{\text{global}},H_{\text{block}}\right)\\ S_{\text{new}}=\max\left(S_{\text{global}},S_{\text{block}}\right)\\ V_{\text{new}}=\max\left(V_{\text{global}},V_{\text{block}}\right) \end{array}\right\}. \end{array}$$

The matrix of all the reserved pixels is the image we finally hope to output. Note here that, for the value of *V*, we also choose a more significant value instead of suppressing it, because this *V* here is different from SR regions that we want to eliminate in this paper. Here, we assume that SR regions have been eliminated, so the value of *V* more affects the brightness of the whole image. Moreover, appropriately increasing the contrast between light and shade can enhance the stereoscopy and the image's visual effect.

## 4. Results

Our experiment is divided into three sections.  In Section 4.1, we set and adjust several essential parameters in eliminating SR regions.  In Section 4.2, we evaluate the effect of inpainting, respectively. Finally, we invite clinicians to conduct clinical evaluation and verification in Section 4.3. All sections involving computer processing are performed on Matlab2018b. The CPU is Intel i7-8700K (3.20 GHz), and the memory is 8.00 GB.

### 4.1. Parameters Setting

In this section, we discuss the settings of several important parameters to study their impact on performance. 150 image samples (Normal, CIN1, CIN2, CIN3, Cancer, 30 in each kind) from Fujian Provincial Maternity and Children's Hospital are selected for verification. The patient information in images is processed for concealment.

#### 4.1.1. Block Numbers

An innovation of this paper is the integration of global and local information, so the regulation of local scope has become a fundamental research problem of this method. In this paper, we mainly deal with local information in the form of blocks, so the determination of the local scope is controlled by the number of blocks. Under the condition of ensuring that other parameters are the same, we conduct five sets of experiments with the number of blocks of 1, 4, 9, 16, and 25 on the colposcopic image and compare the effects of detection and inpainting in turn.

As shown in Figure 6, the first column is the original image and its SR regions mask. The following columns are SR regions detected in combination with different block numbers and corresponding inpainted images. In order to enhance the readability, we have also labelled the details in the figure.

#### 4.1.2. The Coefficient of Local Detection

In the local processing, we choose a simple brightness threshold of the color image. The threshold value directly affects the positioning of SR regions during the local processing and then affects their subsequent inpainting.

As mentioned above, our local detection is controlled by the brightness *y*. Therefore, *y* is treated with four different coefficients of 1.0, 1.1, 1.2, and 1.3, respectively, when the other parameters are the same. The corresponding results of detection are shown in Figure 7. Since the direct effect of this coefficient on inpainting is not obvious, here is not the comparison of inpainting. Similarly, the individual details are marked in the figure.

### 4.2. Inpainting Evaluation

To evaluate the inpainting effect, we first show eliminating results of different lesion grades in our colposcopic image dataset and then extract some literature Atlas to compare several processing methods' subjective visual evaluation grades.

#### 4.2.1. The Preliminary Results

This section shows some experimental results to intuitively reflect the processing effect of our method in different grades of colposcopic images in this paper. As shown in Figure 8, images of different categories are ranked in row order, namely, Normal, CIN1, CIN2, CIN3, and cancer from top to bottom, with an example for each category. From left to right, the sequence from left to right is the resulting image of the original image, Arnold's method, Criminisi's method, the simple combination of the former two methods (Global A + C), and our proposed method integrated global and local information.

#### 4.2.2. Subjective Visual Evaluation

In clinical practice, colposcopic images have no ground truth without SR regions in the real sense, so an objective quantitative evaluation cannot be effectively carried out. Thus, we construct an independent user study to provide honest feedback and quantify subjective evaluation.

Firstly, from 16 pieces of literature [17, 18, 21–23, 25, 26, 28, 31, 32, 34–39] concerning SR elimination from endoscopic images, we extracted 50 images accompanied by their corresponding result images as a new dataset, called Ref_set. Due to the limited research specializing in SR regions elimination of colposcopic images, we extended the images to a broader range of endoscopic images, including some colonoscopic and laparoscopic images. Then, four comparison sets were generated from Ref_set using four methods, including Arnold's method, Criminisi's method, the simple combination of the former two methods, and our proposed method integrated global and local information. Moreover, the result images in those pieces of literature were taken as another comparison set (Ref results), so a total of five comparison sets were used for subjective visual evaluation. Next, we invited 10 testers with basic knowledge of medical anatomy (Group 1) and 10 testers with experience in computer image processing (Group 2). They were required to perform a subjective visual evaluation for each image independently according to their own needs and feelings. The only instruction we gave during the evaluation is as follows: based on SR inpainting, comprehensive visual perception should be used to make a quality rating (1 represents the worst quality, 5 represents the best quality). Finally, we make a statistical analysis of the evaluation results.

The average scores of the 1000 trials are shown in Table 1, and the specific results of the two kinds of participants are separately analyzed. In Figure 9, we also offer the corresponding scatter plots of the five processing methods and the average score of each participant.

### 4.3. Clinical Test

The ultimate goal of medical image processing is to help clinicians improve diagnosis efficiency, so we also perform clinical verification on our method in this paper.

Firstly, we select 300 colposcopic images, including 65 normal or inflammatory samples, 65 CIN1 samples, 60 CIN2 samples, 60 CIN3 samples, and 50 cervical cancer samples. Next, SR regions are eliminated by the proposed method. Then, we randomly mix 300 original images and 300 inpainting images with no SR regions to form an evaluation dataset containing 600 images. Finally, we invite 6 colposcopy physicians to make the independent diagnosis.

In the analysis results, we reseparate the original images from the inpainting images and calculate the accuracy of each physician's diagnosis of colposcopic images before and after eliminating SR regions. In addition, based on the practical clinical significance, we conduct two kinds of classifications: two categories (Normal & Lesion) and four categories (Normal & LSIL & HSIL & Cancer). The statistical results are shown in Table 2. It can be seen that, after eliminating SR regions of colposcopic images, the overall accuracy of physicians is improved to a certain extent. The accuracy of the highest one is increased by 5%. The results of the two categories mainly show positive effects, while the negative impact is slightly increased in the more refined four categories.

## 5. Discussion

This paper proposes a method to eliminate SR regions of colposcopic images and conduct various experimental tests on its performance in many aspects.

In the parameters section, we explore the number of blocks and local detection coefficients. In Figure 6, we focus on the comparison of several details of the labels. When the number of blocks is 9 and 16, the overall image restoration effect is better, but the restoration of 9 blocks takes less time. Therefore, for our dataset, in combination with the time and final effect, we believe that the performance is the best when the number of blocks is set to 9. As shown in Figure 7, with the continuous increase of the coefficient, the detected region decreases, and some SR regions with scattered distribution are lost. However, the refinement of the details is more in line with the actual SR regions positioning in the image, such as the region circled by the ellipse in the lower right corner. To balance the above two points, we apply a local detection coefficient of 1.2 to our dataset.

The overall effect of eliminating SR regions in colposcopic images is verified by subjective visual evaluation from the computer and medical perspectives to make up for the defect of comparative evaluation of no ground truth as much as possible. The evaluation results in Table 1 show that our method of integrating global and local information for eliminating SR regions in colposcopic images has the best performance from the computer processing perspective. And the effect is the same as that in the published literature from a medical standpoint. Overall, the proposed method has sound visual effects. In Figure 9, the red dots representing the proposed method are kept at the top of each group. In a sense, this small-scale experiment makes up for the lack of ground truth to make the effective quantitative evaluation in eliminating SR regions in the colposcopic image and provides additional support for our method of integrating global and local information to eliminate SR regions.

As for clinical testing, in response to the increase in the negative impact of the four categories, we further conduct statistics on each of the four categories' accuracy and observe that the negative effect is concentrated in the Cancer category. We have feedback communication with the physicians about this result and learned that, to avoid overdiagnosis in clinical diagnosis, the physicians would maintain a conservative attitude toward a diagnosis in most cases. Ultimately, the pathological biopsy result is taken as the gold standard. Physicians often tend to make a conservative diagnosis for the images after eliminating SR regions due to insufficient brightness. This feedback also arouses our thinking. Besides the improvement of the method, the clinical application of SR elimination from colposcopic images should focus on the needs of physicians. In the process of colposcopy, when physicians find that the SR regions in the collected image interfere with the lesion diagnosis, they can select the operation of SR elimination in real-time and can also perform the comparison before and after eliminating SR regions, thus increasing the accuracy of the clinician's diagnosis.

In addition, some endoscopic datasets are involved in the detection and inpainting evaluations in this paper. The relevant evaluation results are good, proving that the method has a long-lasting effect not only for the targeted restoration of SR regions in colposcopic images, but also for other similar endoscopic images.

## 6. Conclusions

We introduce a method of eliminating SR regions by integrating the global and local information of colposcopic images in this paper. Our method preserves and constructs the texture and structure information in SR regions as much as possible, thus increasing the visual observability of the image. Many results have been achieved in computer and clinical tests. In contrast to experiments on eliminating SR regions in endoscopic images, our method still has good performance, so it has potential value for similar visual tasks of this kind of image.

## Figures and Tables

**Figure 1:** Features of cervical lesions under colposcopy.

**Figure 2:** The flowchart of the proposed method.

**Figure 3:** Data samples.

**Figure 4:** The flowchart of global SR detection.

**Figure 5:** The model of exemplar-based method for SR regions inpainting.

**Figure 6:** Comparation of the number of blocks.

**Figure 7:** Comparison of local detection threshold coefficients.

**Figure 8:** Experimental results of different grades of lesions.

**Figure 9:** Scatter plot of subjective visual evaluation.

**Table 1:** Subjective visual evaluation score.

	Arnold's	Criminisi's	Ref results	Global A + C	The proposed
Group 1	3.28	3.43	**3.63**	3.56	**3.63**
Group 2	2.47	2.81	3.41	3.45	**3.48**
Average	2.88	3.12	3.52	3.51	**3.55**

Bold values represent the best data in each group.

**Table 2:** Accuracy of clinical evaluation results (%).

Physician	Normal & lesion			Normal & LSIL & HSIL & cancer		
	Original (%)	No SR (%)	Influence (%)	Original (%)	No SR (%)	Influence (%)
1	76.67	79.00	2.33	48.33	51.67	3.34
2	69.67	71.00	1.33	48.00	50.00	2.00
3	60.67	61.67	1.00	47.00	44.67	−2.33
4	67.00	66.33	−0.67	46.33	45.67	−0.66
5	68.00	72.33	4.33	40.67	45.67	**5.00**
6	47.00	51.00	4.00	28.33	29.67	1.34
Average	64.83	66.89	2.06	43.11	44.56	1.44

Bold values represent the best data in the evaluation.

## Data Availability

The processed data required to reproduce these findings cannot be shared at this time as the data also form part of an ongoing study.
